# Effects of Carvedilol on Blood Pressure, Blood Sugar, and Blood Lipids in Elderly Patients with Refractory Hypertension

This article has been retracted.

**DOI:** 10.1155/2022/7889024

**Published:** 2022-07-27

**Authors:** Wen Zhang, Guiming Deng, Jia Hu, Ran Yan, Junliu Hu, Jianmin Fan

**Affiliations:** ^1^The First Hospital of Hunan University of Chinese Medicine, Department of Geriatrics, No. 95 Shaoshan Middle Road, Yuhua District, Changsha City, Hunan Province, China; ^2^Hunan University of Chinese Medicine, Graduate School, Xiangzui Road, Yuelu District, Changsha City, Hunan Province, China; ^3^Hunan University of Chinese Medicine, School of Traditional Chinese Medicine, Xiangzui Road, Yuelu District, Changsha City, Hunan Province, China; ^4^The First Hospital of Hunan University of Chinese Medicine, Department of Cardiovascular Diseases, No. 95 Shaoshan Middle Road, Yuhua District, Changsha City, Hunan Province, China

## Abstract

Refractory hypertension seriously affects the life safety of patients. To investigate the effect of carvedilol combined with conventional antihypertensive therapy on blood pressure, blood sugar, blood lipids, and cardiovascular and cerebrovascular complications in elderly patients with refractory hypertension, a total of 80 elderly patients with refractory hypertension who were admitted from June 2019 to September 2021 were selected as the retrospective research objects and divided into the observation group and the control group according to the random number table method, 40 cases in each group, and the control group received conventional antihypertensive therapy. On this basis, the observation group was treated with carvedilol, and the effects of blood pressure, blood sugar, blood lipids, and cardiovascular and cerebrovascular complications were analyzed in the two groups. After treatment, the systolic blood pressure, diastolic blood pressure, adrenal medulla (AM), and endothelin (ET) of the observation group were significantly lower than those of the control group, but the heart rate and NO of the observation group were significantly higher than those of the control group. After treatment, the fasting blood glucose, insulin, triacylglycerol (TG), cholesterol (CHO), and low-density lipoprotein (LDL-C) of the observation group were significantly higher than those of the control group, but the ISI and HDL-C of the observation group were significantly lower than those of the control group. After treatment, the levels of IL-1*β*, IL-6, TNF-*α*, UAER, BUN, and SCr in the observation group were significantly lower than those in the control group. The TC of the observation group was lower than that of the control group. Combination therapy has a remarkably stable, sustained, and safe antihypertensive effect on patients with refractory hypertension.

## 1. Introduction

Refractory hypertension is defined as the application of a reasonably tolerable adequate dose of >3 antihypertensive drugs on the basis of lifestyle improvement, treatment for >1 month and still not achieving the blood pressure standard, or taking >4 antihypertensive drugs for effective blood pressure control [1–3]. The prevalence of refractory hypertension has increased gradually over a 20-year period, which may be related to the increased awareness, treatment, and management of hypertension in the United States and certainly to the increasing prevalence of aging and obesity [4]. We speculate that the prevalence of true refractory hypertension may not be high and that many patients may have pseudorefractory hypertension due to irrational medication use and poor compliance [5]. Carvedilol is a nonselective *β*-blocker that blocks *β* receptors comprehensively and also selectively blocks *α*1 receptors, without endogenous sympathomimetic activity or peripheral *β* agonism [6]. Poor control of blood pressure in refractory hypertension can easily lead to target organ damage, leading to more serious consequences.

Carvedilol, as a third-generation *β*-blocker, has characteristics unmatched by other receptor blockers and is widely used in the treatment of hypertension, congestive heart failure, and coronary artery disease, with positive efficacy [7]. Some studies have shown that carvedilol can subside left ventricular hypertrophy and improve diastolic function in hypertensive patients [8]. There are few reports in the literature on the therapeutic effects of carvedilol with various antihypertensive drugs, and this paper examines the effects of carvedilol combined with conventional antihypertensive therapy on blood pressure, glucose, lipids, and cardiovascular complications in elderly patients with refractory hypertension.

## 2. Material and Methods

### 2.1. Research Object

Eighty cases of elderly patients with refractory hypertension admitted from June 2019 to September 2021 were selected for the retrospective study and were divided into 40 cases each in the observation and comparison groups according to the random number table method. Hypertension was diagnosed according to the criteria in the Chinese Guidelines for the Prevention and Treatment of Hypertension (2010 edition) [9], with an office systolic blood pressure ≥ 140 mmHg and/or diastolic blood pressure ≥ 90 mmHg, or taking antihypertensive drugs as hypertension: 140-159/90-99 mmHg as grade 1 hypertension, 160-179/100-109 mmHg as grade 2 hypertension, and ≥180/110 mmHg as grade 3 hypertension. Systolic blood pressure < 140 mmHg and diastolic blood pressure ≥ 90 mmHg were defined as pure diastolic hypertension, systolic blood pressure ≥ 140 mmHg and diastolic blood pressure < 90 mmHg were defined as pure systolic hypertension, and systolic blood pressure ≥ 140 mmHg and diastolic blood pressure ≥ 90 mmHg were defined as dual systolic-diastolic hypertension. Refractory hypertension was defined as office blood pressure ≥ 140/90 mmHg after taking ≥3 antihypertensive drugs (including a diuretic) or office blood pressure < 140/90 mmHg, but ≥4 antihypertensive drugs were required. The hypertension awareness rate was defined as the percentage of the total number of hypertensive patients who knew they had hypertension; the hypertension treatment rate was defined as the percentage of the total number of hypertensive patients who were taking antihypertensive drugs in the past two weeks; the hypertension control rate was defined as the percentage of the total number of hypertensive patients whose blood pressure was controlled to the target value (systolic blood pressure < 140 mmHg and diastolic blood pressure < 90 mmHg).

### 2.2. Inclusion and Exclusion Criteria

Inclusion criteria: (1) those with good compliance and able to cooperate with medical staff to complete our study; (2) those without congestive heart failure, acute myocarditis, acute myocardial infarction, diabetes mellitus, etc.; (3) those without history of surgery and other infectious diseases. Exclusion criteria: (1) severe diabetes mellitus with uncontrollable symptoms, infection or blood transfusion within 3 months, other chronic diseases such as malignancy, and change of treatment plan within 3 months; (2) those who do not actively cooperate with treatment, history of blood transfusion, and major trauma and surgery in the last 3 months; (3) secondary hypertension, liver and kidney dysfunction, and history of allergy to the drugs used in our study.

### 2.3. Methods

In the control group, conventional antihypertensive therapy was administered, with 80 mg/d of gelsartan (produced by Beijing Novartis Pharmaceutical Co., Ltd.) and 1 tablet/d of compound amiloride hydrochloride (produced by Jiangsu Tianhe Pharmaceutical Co., Ltd.) The first 4 weeks were the transition period of the drug, and after 4 weeks, if the blood pressure decreased to an effective level, the drug was taken for another 4 weeks at the original dose, and the blood pressure was reduced and maintained if it was stable, and the blood pressure was <120/80 mmHg and accompanied by dizziness. For those with blood pressure < 120/80 mmHg and dizziness, the compound amiloride hydrochloride could be reduced and stopped. However, the observation group was treated with carvedilol, taking 80 mg/d of gelsartan (produced by Beijing Novartis Pharmaceutical Co., Ltd.); 12.5 mg/d of carvedilol (produced by Shanghai Roche Pharmaceutical Co., Ltd.), and if tolerated, the dose was increased to 25 mg/d after two days; and 1 tablet/d of compound amiloride hydrochloride (produced by Jiangsu Tianhe Pharmaceutical Co., Ltd.). The first 4 weeks were the transition period of the drug, and after 4 weeks, if the blood pressure decreased to an effective level, then the dose was reduced again. If the blood pressure decreases effectively, the drug will be taken for another 4 weeks at the original dose; if the blood pressure is stable, the dose will be reduced and maintained; if the blood pressure is <120/80 mmHg and accompanied by dizziness, the compound amiloride hydrochloride can be reduced and stopped.

### 2.4. Observation Index

Inflammatory factors and endothelial function factors: 5 ml of fasting venous blood was drawn before treatment and 1 month after treatment, respectively, and centrifuged at 3000 r/min for 5 min, and the supernatant liquid was placed in EP tubes and stored at -70°C. Serum interleukin- (IL-) 1B and IL-6 were detected in EP tubes by enzyme-linked immunosorbent assay (ELISA), and the kits were purchased from Shanghai ELISA Biotechnology Co. Plasma adrenal medulla (AM) and endothelin (ET) were detected by Beckman luminescence immunoassay, and nitric oxide (NO) was detected by nitrate reductase assay. The 24 h urinary protein excretion rate (UAER), serum creatinine (SCr), blood urea ammonia (BUN), total cholesterol (TC), and triacylglycerol (TG) were measured before and after treatment, and occasional blood pressure (OBP) and ambulatory blood pressure (ABP) were monitored. In all cases, the sitting blood pressure after 15 minutes of rest was measured three times with a mercury column sphygmomanometer on the day of treatment initiation and at the end of treatment, and the mean values were taken. Blood glucose and lipid were measured by American Beckman CX4 biochemical instrument, insulin was measured by radioimmunoassay (the kit was provided by the Reagent Research Institute of China Isotope Company), and the insulin sensitivity index (ISI) was calculated by the formula ln [1/(fasting blood glucose × fasting insulin)].

### 2.5. Statistical Analysis

All statistical data in this study were entered into Excel software by the first author and the corresponding author, respectively, and the statistical processing software was SPSS 25.0 for calculation. Repeated measures analysis of variance between groups was used to measure the measurement expressed as mean ± standard deviation (*X* ± *S*) material. Count data expressed as a percentage (%) were tested by *χ*^2^. Included data that did not conform to a normal distribution were described by *M* (QR), using the Mann–Whitney test. All statistical tests were two-sided probability tests. The statistical significance was *P* < 0.05.

## 3. Results

### 3.1. Comparison of Baseline Data

The mean age, gender, disease duration, and weight of the patients in the observation group were not significantly different from those in the comparison group, and the comparative differences were not statistically significant (*P* > 0.05). See Table 1.

### 3.2. Comparison of Blood Pressure-Related Indicators

There was no statistical significance in the blood pressure-related indexes before treatment (*P* > 0.05). After treatment, the systolic blood pressure, diastolic blood pressure, AM, and ET of the observation group were significantly lower than those of the control group, but the heart rate and NO of the observation group were significantly higher than those of the control group, and the differences were statistically significant (*P* < 0.05). See Figure 1.

### 3.3. Blood Lipid and Blood Sugar Comparison

After treatment, the fasting blood glucose, insulin, TG, CHO, and LDL-C of the observation group were significantly higher than those of the control group, but the ISI and HDL-C of the observation group were significantly lower than those of the control group, and the differences were statistically significant (*P* < 0.05). See Figure 2.

### 3.4. Serum Index Comparison

There was no significant difference in serum indexes between the two groups before treatment (*P* > 0.05). After treatment, the levels of IL-1*β*, IL-6, TNF-*α*, UAER, BUN, and SCr in the observation group were significantly lower than those in the control group. The TC of the observation group was lower than that of the control group, and the difference was statistically significant (*P* < 0.05). See Figure 3.

## 4. Discussion

Refractory hypertension is a common clinical condition that is more difficult to treat. Carvedilol is a nonselective *β*-blocker, which can fully block *β* receptors and also selectively block *α*1 receptors without endogenous sympathomimetic activity and peripheral *β* agonism [10]. Carvedilol, as a third-generation *β*-blocker, has characteristics unmatched by other *β*2-blockers and is widely used in the treatment of hypertension, congestive heart failure, and coronary artery disease with proven efficacy [11]. Some studies have shown that carvedilol can subside left ventricular hypertrophy and improve diastolic function in hypertensive patients. In contrast, spironolactone, as a potassium-preserving diuretic, has a weak diuretic and antihypertensive effect [12]. However, recent studies have found that spironolactone not only has potassium-preserving and sodium-removing effects but also has protective effects on the cardiovascular system when combined with other antihypertensive drugs as an aldosterone antagonist, which can further block RAAS to improve the antihypertensive effect [13].

Our study found that the systolic blood pressure, diastolic blood pressure, AM, and ET in the observation group were significantly lower than those in the comparison group after treatment; however, the heart rate and NO in the observation group were significantly higher than those in the comparison group, and the comparative differences were all statistically significant. IL-1*β*, IL-6, TNF-*α*, UAER, BUN, and SCr in the observation group were significantly lower than those in the comparison group after treatment; however, TC in the observation group were lower than those in the comparison group, and the comparative differences were all statistically significant. It indicates that the combination therapy has a significantly smooth, sustained, and safe antihypertensive effect on patients with refractory hypertension. The long-term hypertensive state of patients can lead to myocardial remodeling and direct damage to vascular endothelial cells, which can even cause chronic heart failure [14]. Among them, various inflammatory cytokines and endothelial function indicators play an important regulatory role in disease progression; for example, IL-1*β*, IL-6, and TNF-*α* exacerbate heart failure by regulating cardiovascular function in patients [15]. Therefore, it is crucial to prevent or delay the process of heart failure in the course of antihypertension [16]. Studies have shown that carvedilol blocks B receptors while also exerting antioxidant, anti-inflammatory, and antiapoptotic effects, thereby inhibiting NF-*κ*B activity, suppressing the secretion of inflammatory factors by inflammatory cells, reducing the invasion of cardiomyocytes, and improving cardiac function [17]. This study showed that both can effectively improve inflammatory factor levels and endothelial function with similar effects. Studies in the literature have shown that benazepril, amlodipine, and irbesartan all improve endothelial function in patients, i.e., by increasing NO levels and decreasing AM and ET levels, thereby improving vascular endothelial function, delaying target organ damage, and reducing the risk of cardiovascular and cerebrovascular events [18]. The improvement of endothelial function can effectively respond to the improvement of blood pressure variability in patients with hypertension, thus indicating a stable antihypertensive effect [19]. Current studies confirm that the onset and development of hypertension are associated with functional and structural changes in endothelial cells, and the hypertensive state may further aggravate the functional and structural damage of vascular endothelial cells and vascular smooth muscle cells [20]. Among them, plasma ET and NO are a pair of vasoactive substances with antagonistic effects synthesized by vascular endothelial cells, which have an important role in the regulation of vascular smooth muscle function and vascular tone [21]. NO is an atomic group produced by L-arginine as a result of endothelial cell stimulation, which enters vascular smooth muscle cells to activate endoguanylate cyclase and increase intracellular CGMP content [22]. This leads to vascular smooth muscle diastole, inhibition of platelet agglutination, inhibition of endocytosis, and thus inhibition of thrombus formation, and the above effects make it useful in hypertension [23]. ET is a vasoactive peptide consisting of 21 amino acids and is the most potent long-acting vasoconstrictor known [24]. The possible mechanisms of ET involvement in the pathogenesis of EH are as follows: specific binding of ET to vascular smooth muscle on ET activates the renin-angiotensin-aldosterone system, causing a strong vasoconstrictor effect of angiotensin I. ET increases vascular responsiveness to other vasoconstrictors such as endogenous and exogenous norepinephrine substances [25]. ET promotes vascular smooth muscle cell proliferation and hypertrophy, resulting in narrowing of the lumen, thickening of the vessel wall, and increased peripheral resistance, and activation of phospholipase A2, which produces thromboxane A2, can further enhance vasoconstriction and increase blood pressure [26]. The increase in blood pressure increases the shear stress on the vessel wall and promotes the expression of ET-mRNA, and EH in turn can aggravate endothelial damage and increase endothelial dysfunction, with impaired production of diastolic substances such as nitric oxide (NO) and prostacyclin (PGL2) and increased release of thromboxane A2, along with massive secretion of ET [27].

Our study found that fasting glucose, insulin, TG, CHO, and LDL-C were significantly higher in the observation group than in the comparison group; however, ISI and HDL-C were significantly lower in the observation group than in the comparison group, and the comparative differences were all statistically significant. We know that traditional *β*-blockers can lead to an increase in TG and CHO levels as well as abnormalities in glucose tolerance and increased insulin resistance while exerting therapeutic effects [28]. Therefore, improving 3-blockers and improving lipid and glucose metabolism become essential. Consideration is mainly due to the fact that carvedilol is a nonselective *β*-blocker that selectively blocks the receptors along with the full range of B receptors [29]. At the same time, carvedilol is able to increase insulin sensitivity and improve lipid and glucose metabolism in general, which is related to the receptor blocker effect of carvedilol as well as elevating lipid oxidase activity and regulating disordered lipid and glucose metabolism [30]. Thus, carvedilol is effective in lowering blood pressure while having effects that are not found in other *β*-blockers, which improve insulin sensitivity [31].

This study was a case-control study, not a randomized controlled trial, and was not blinded, so there is still a certain risk of bias; the sample size included was small, there is still a need to subsequently increase the sample size and conduct multicenter clinical studies, the clinical follow-up period was short, and long-term clinical follow-up observations are still needed. In conclusion, the combination therapy had significant smooth, sustained, and safe antihypertensive effects on refractory hypertensive patients, with similar effects on endothelial function and control of various inflammatory factors and consistent recent efficacy, which is worth further promotion.

## Figures and Tables

**Figure 1:** Comparison of blood pressure-related indicators. The data of blood pressure-related indicators of our study were entered into Excel software by the first and corresponding authors, and the statistical processing software was SPSS 25.0 for calculation. Using the mean ± standard deviation (*X* ± *S*) representation using the independent sample *t*-test.

**Figure 2:** Blood lipid and blood sugar comparison. Blood lipid and blood sugar comparison data from our study were entered into Excel software by the first and corresponding authors, and statistical processing software was SPSS 25.0 for calculation. The mean ± standard deviation (*X* ± *S*) was used to express the results using independent sample *t*-test.

**Figure 3:** Serum index comparison. The comparative serum index data of our study were entered into Excel software by the first and corresponding authors, and the statistical processing software was SPSS 25.0 for calculation. Using the mean ± standard deviation (*X* ± *S*) to indicate the use of independent sample *t*-test.

**Table 1:** Comparison of baseline information between the two groups of patients ($\bar{X}\pm S$).

Group	Average age (years)	Gender (male/female)	Duration of disease (years)	Body weight (kg)
Comparison group (40)	60.90 ± 1.71	24/26	3.05 ± 1.23	62.35 ± 2.10
Observation group (40)	61.10 ± 1.62	23/27	2.40 ± 2.03	60.10 ± 1.10
*t*	0.377	0.731	0.763	2.107
*P*	0.051	0.067	0.091	0.079

## Data Availability

The datasets used and analyzed during the current study are available from the corresponding author upon reasonable request.
